# Optimized Fuzzy C-Means Algorithm-Based Coronal Magnetic Resonance Imaging Scanning in Tracheal Foreign Bodies of Children

**DOI:** 10.1155/2021/5678994

**Published:** 2021-07-07

**Authors:** Lan Jin, Ke Chang

**Affiliations:** Department of Pediatrics, Hospital of Chengdu University of Traditional Chinese Medicine, Chengdu 610072, Sichuan, China

## Abstract

In order to provide theoretical support for clinical diagnosis, the diagnostic value of the optimized fuzzy C-means (FCM) algorithm combined with coronal magnetic resonance imaging (MRI) scan was investigated in the diagnosis of tracheal foreign bodies in children. The anisotropic filtering was applied to optimize the traditional FCM algorithm, so as to construct a new MRI image segmentation algorithm, namely, AFFCM algorithm. Then, the traditional FCM algorithm, the FCM algorithm based on the kernel function (KFCM), and the FCM algorithm based on the spatial neighborhood information (RFCM) were introduced for comparison with the AFFCM. 28 children diagnosed with foreign bodies in the trachea were selected for MRI diagnosis, and AFFCM was used for segmentation. The partition coefficient, segmentation entropy, and the correlation degree between classes after fuzzy division of the four algorithms were recorded, and the location and distribution of foreign bodies in the trachea and the types of foreign bodies were also collected. Besides, the MRI scanning and chest X-rays of the children with foreign bodies in the trachea should also be recorded in terms of the positive rate, diagnosis rate, and indirect signs. The class division coefficient and interclass correlation degree after fuzzy division of AFFCM were markedly greater than those of FCM, KFCM, and RFCM (*P* < 0.05), while the segmentation entropy of AFFCM was less sharp than the entropies of FCM, KFCM, and RFCM (*P* < 0.05). Among the 28 children, there were 5 cases with foreign bodies in the trachea (17.86%), 10 cases in the left bronchus (35.71%), and 13 cases in the right bronchus (46.43%). Among the foreign body types, there were 10 cases of melon seeds (35.71%), 6 cases of peanuts (21.43%), and 5 cases of beans (17.86%). The positive rate (89.29%) and diagnosis rate (96.43%) of MRI for bronchial foreign bodies increased obviously in contrast to the rates of X-ray chest radiographs (57.14% and 67.86%) (*P* < 0.05). Therefore, it was indicated that AFFCM showed higher partition coefficient value, lower segmentation entropy, larger similarity among classes, and better image segmentation effect. Furthermore, AFFCM-based coronal MRI scan had a higher positive rate and diagnosis rate for children's tracheal foreign bodies, and the main signs were emphysema and atelectasis.

## 1. Introduction

Tracheal foreign bodies in children refer to foreign bodies entering the airway, causing airway blockage. In mild cases, it can result in lung damage, and, in severe cases, suffocation death is more common in children below 5 years of age [1]. The most common manifestations of foreign bodies in the trachea of children are severe coughing, suffocation, nausea, excessive phlegm, and difficulty breathing [2]. If it is not treated in time, it will easily lead to suffocation, atelectasis, recurrent pneumonia, which will not heal for a long time, and even death in severe cases. Therefore, timely diagnosis of foreign bodies in the trachea of children is necessary. The clinical diagnosis methods for foreign bodies in the trachea of children mainly include X-ray, ordinary computed tomography (CT), and multislice spiral CT [3, 4]. When diagnosing atypical foreign bodies in the trachea of infants and young children, it is necessary to use X-rays for chest plain radiographs and fluoroscopy to determine the presence of foreign bodies through indirect signs. However, when the imaging manifestations such as pulmonary obstruction, pulmonary block shadows, and atelectasis occur, it is easy to be misdiagnosed as bronchial pneumonia, bronchial lung cancer, bronchial asthma, and other diseases, and the misdiagnosis rate is high [5]. Ordinary CT axial images increase the detection rate of foreign bodies, and the display clarity of indirect lung signs is better than X-ray, but it has the disadvantages of slow scanning speed, only presenting axial images, and easy to miss small foreign bodies. Multislice spiral CT is developed based on common CT technology, which greatly shortens the scanning time, and has higher resolution and image clarity, but it does not perform well in soft tissue display and needs further improvement. MRI examination is an auxiliary examination method that is extensively applied in clinical practice. It is different from X-ray film, CT, and other methods, which can accurately locate the lesion and make qualitative diagnosis of the lesion. It is mainly suitable for soft tissues, bones and joints, nervous system, and chest and abdomen [6, 7].

Due to the uncertainty of the gray scale and geometric shape of the digital image, it is quite difficult to use the digital image. Therefore, it is necessary to apply fuzzy theory and robust algorithm to process these digital images [8]. Among them, fuzzy C-means (FCM) is the most widely used objective function-based fuzzy clustering method in daily life applications. It occupies a key position in the field of image segmentation and can be used for gray image or color image segmentation [9]. FCM can obtain the minimum value of the objective function through an iterative optimization method, thereby updating the membership of the elements in the sample set and finally obtaining the optimal cluster center [10, 11]. However, FCM also has some inherent shortcomings. For example, FCM will become very sensitive and affect the accuracy of the segmentation results when some sample images with natural noise are encountered. Based on this, the introduction of anisotropic filtering was considered in this study to optimize the FCM algorithm and apply it to the sagittal MRI image processing of pediatric bronchial foreign bodies.

To sum up, the application of mathematical algorithms and magnetic resonance imaging (MRI) images in the field of medical diagnosis is the focus of the current research. On this basis, anisotropic filtering was employed to optimize the traditional fuzzy clustering method, and a new MRI image segmentation algorithm was constructed in this study. In addition, the traditional fuzzy clustering algorithm, the FCM algorithm based on the kernel function (KFCM), and the rough FCM (RFCM) were also introduced, which were compared with the fuzzy clustering algorithm. 28 pediatric patients diagnosed with foreign bodies in the trachea were selected for MRI diagnosis, and AFFCM was used for segmentation to comprehensively evaluate the diagnostic value of modified FCM combined with coronal MRI scanning in children with foreign bodies in the trachea.

## 2. Materials and Methods

### 2.1. Research Objects

28 child patients, who were hospitalized with foreign bodies in the trachea in the hospital from October 2019 to November 2020, were selected as the research objects in this study. There were 17 males and 11 females, with the age ranging from 5 months to 10 years, and the history of foreign body inhalation ranged from 5 hours to 32 days. This study had been approved by the ethics committee of the hospital, and the family members of the child patients included in the study were known and signed the informed consent forms.

The inclusion criteria were defined to include child patients who were diagnosed with foreign bodies in the trachea, signed the informed consent forms, and had no contraindications to MRI scanning.

The exclusion criteria were defined to include child patients who had received relevant treatment, withdrew from the experiment halfway, and had other lung diseases.

### 2.2. Coronary MRI and X-Ray Scanning

The requirements of MRI scanning were as follows: A 3.0 T superconducting magnetic resonance MAGNETOM Skyra imaging system (produced by Siemens, Germany) was adopted in this study to scan the child patients. First, each child patient was placed in a supine position and underwent the cross-sectional and sagittal positioning scanning. Besides, a coronal scanning was performed with the child's trachea and bronchus bifurcation as the center to obtain the coronal T1-weighted imagining (T1WI) of the self-cyclotron wave sequence. The scanning parameters included repetition time (TR) of 400 ms, echo time (TE) of 15 ms, and layer thickness of 5 mm.

The requirements of chest X-ray were shown in the following. In this study, PHILIPS DR machine (produced by Royal Philips, Netherlands) was used for X-ray examination, and each child patient was placed in a supine position, inhaled, and taken X-ray after the chest was in the center.

### 2.3. FCM Based on Anisotropic Filtering Optimization

FCM can minimize the objective function through the iterative calculation of the membership matrix and clustering center, and then the data sample set is partitioned by defuzzing operation according to the membership matrix [4]. When FCM is applied to image segmentation, all pixels on the image to be segmented are the sample set of data, and its objective function can be expressed as follows:

(1) $$\begin{array}{c} G_{\alpha }\left(W,Z\right)=\sum_{i=1}^{n}\sum_{j=1}^{s}{\left(w_{ji}\right)}^{\alpha }l^{2}\left(x_{i},z\right), \end{array}$$

(2) $$\begin{array}{c} \sum_{j=1}^{s}\left(w_{ji}\right)=1. \end{array}$$

In equations (1) and (2), *s* represents the number of clusters, *n* stands for the number of pixels, *W* expresses the value of the membership function, *S*=(*w*_*ji*_)_*s*×*n*_, *Z* indicates the central value of all clusters, *Z*=(*z*_1_, *z*_2_,…*z*_*n*_), *x*_*i*_ means the gray value of the image pixel, *α* represents the fuzzy weighted index, and *l*^2^(*x*_*i*_, *z*) indicates the square of the error within the class. Then, the Lagrangian multiplier method is introduced to solve equations (1) and (2):

(3) $$\begin{array}{c} H=\sum_{j=1}^{s}{\left(w_{ji}\right)}^{\alpha }l_{ji}^{2}+\beta \left(1-\sum_{j=1}^{s}w_{ji}\right). \end{array}$$

In equation (3), *H* represents the Lagrangian multiplier solution, and *α* and *β* stand for the parameters. Then, the necessary conditions for the optimization of the Lagrangian equation should be the following:

(4) $$\begin{array}{c} \frac{\partial H}{\partial \beta }=1-\sum_{j=1}^{s}w_{ji}=0, \end{array}$$

(5) $$\begin{array}{c} \frac{\partial H}{\partial w_{ji}}=\alpha {\left(w_{ji}\right)}^{\alpha -1}{\left(l_{ji}\right)}^{2}-\beta =0. \end{array}$$

From equation (4), the following equation can be obtained:

(6) $$\begin{array}{c} w_{ji}={\left[\frac{\beta }{\alpha {\left(l_{ji}\right)}^{2}}\right]}^{\left(1/\alpha -1\right)}. \end{array}$$

Equation (5) is substituted into equation (2), so as to obtain the two following equations:

(7) $$\begin{array}{c} \sum_{j=1}^{s}w_{ji}={\left(\frac{\beta }{\alpha }\right)}^{1/\alpha -1}\left\{\sum_{j=1}^{s}\left[{\frac{1}{{\left(l_{ji}\right)}^{2}}}^{1/\alpha -1}\right]\right\}=1, \end{array}$$

(8) $$\begin{array}{c} {\left(\frac{\beta }{\alpha }\right)}^{{1/}^{\alpha -1}}=\frac{1}{\sum_{j=1}^{s}{\left[1/{\left(l_{ji}\right)}^{2}\right]}^{1/\alpha -1}}. \end{array}$$

Equation (9) can be obtained by substituting equation (8) into equation (5).

(9) $$\begin{array}{c} w_{ji}=\frac{1}{\sum_{p=1}^{s}{\left[l_{ji}/l_{jp}\right]}^{2/\alpha -1}}. \end{array}$$

Then, *G*_*α*_(*W*, *Z*) is made to be the minimum membership function value, which can be shown in the following equation:

(10) $$\begin{array}{c} w_{ji}={\left[\frac{\beta }{\alpha {\left(l_{ji}\right)}^{2}}\right]}^{1/\alpha -1}. \end{array}$$

In the same way, *G*_*α*_(*W*, *Z*) is made to be the smallest cluster center value, as shown in the following equation:

(11) $$\begin{array}{c} Z_{i}=\frac{\sum_{i=1}^{n}{\left(w_{ji}\right)}^{\alpha }x_{i}}{\sum_{i=1}^{n}{\left(w_{ji}\right)}^{\alpha }}. \end{array}$$

Therefore, the cluster center and the best classification matrix can be determined by equations (10) and (11) according to the number of cluster categories of the data sample set and the specified sample fuzzy weight. What is more, the defuzzy algorithm [12] is applied to operate the membership matrix to complete the partition effect of samples. However, the standard FCM algorithm does not consider the association of the neighboring pixels of each element when performing image segmentation, which makes the algorithm very sensitive to images with noise. Therefore, the anisotropic filtering method was introduced in this study to denoise the image by anisotropic filtering, and its objective function can be updated as follows:

(12) $$\begin{array}{c} G{}^{*}=\overset{s}{\underset{j=1}{\sum }}\overset{T-1}{\underset{t=0}{\sum }}f_{x}\left(t\right)w_{jt}^{\alpha }{\left\|\Phi \left(x_{t}\right)-\Phi \left(z_{j}\right)\right\|}^{2}+\kappa \overset{s}{\underset{j=1}{\sum }}\overset{T-1}{\underset{t=0}{\sum }}f_{y}\left(t\right)w_{jt}^{\alpha }{\left\|\Phi \left(y_{t}\right)-\Phi \left(z_{j}\right)\right\|}^{2}. \end{array}$$

In equation (12), *t* stands for the gray level in the image, *T* represents the highest gray level in the image, *f*(*t*) means the gray domain histogram statistical function of the image before and after processing, *κ* indicates the coefficient of fuzzy weight correction, *y* represents the gray value of the postprocessing image, and Φ(*x*) represents the kernel function. Φ(*x*) is set as the Gaussian kernel function ([*K*()]), so the following equations can be gotten:

(13) $$\begin{array}{c} {\left\|\Phi \left(x_{i}\right)-\Phi \left(z_{j}\right)\right\|}^{2}=K\left(x,x\right)+K\left(y,y\right)-2K\left(x,y\right), \end{array}$$

(14) $$\begin{array}{c} K\left(x,y\right)=\exp\left(-\frac{{\left\|x-y\right\|}^{2}}{\theta^{2}}\right). \end{array}$$

From equations (13) and (14), the following equation can be obtained:

(15) $$\begin{array}{c} {\left\|\Phi \left(x_{i}\right)-\Phi \left(z_{j}\right)\right\|}^{2}=2\left(1-K\left(x_{i},z_{j}\right)\right). \end{array}$$

Thus, the objective function can be updated as follows:

(16) $$\begin{array}{c} G{}^{*}=\overset{s}{\underset{j=1}{\sum }}\overset{T-1}{\underset{t=0}{\sum }}f_{x}\left(t\right)w_{jt}^{\alpha }\left(1-K\left(x_{i},z_{j}\right)\right)+\kappa \overset{s}{\underset{j=1}{\sum }}\overset{T-1}{\underset{t=0}{\sum }}f_{y}\left(t\right)w_{jt}^{\alpha }\left(1-K\left(y_{i},z_{j}\right)\right). \end{array}$$

The same can be solved to make *G∗*(*W*, *Z*) the minimum membership function value and cluster center value, which can be expressed in the two following equations:

(17) $$\begin{array}{c} w_{ji}=\frac{{\left[f_{x}\left(t\right)\left(1-K\left(x_{i},z_{j}\right)\right)+\beta f_{y}\left(t\right)\left(1-K\left(y_{i},z_{j}\right)\right)\right]}^{1/\alpha -1}}{\sum_{j=1}^{s}\left[f_{x}\left(t\right)\left(1-K\left(x_{i},z_{j}\right)\right)+\beta f_{y}\left(t\right){\left(1-K\left(y_{i},z_{j}\right)\right)}^{1/\alpha -1}\right]}, \end{array}$$

(18) $$\begin{array}{c} Z_{i}=\frac{\sum_{t=0}^{T-1}\left[f_{x}\left(t\right)w_{jt}^{\alpha }K\left(x_{i},z_{j}\right)x_{t}+\beta f_{y}\left(t\right)w_{jt}^{\alpha }K\left(y_{i},z_{j}\right)y_{t}\right]}{\sum_{j=1}^{s}\left[f_{x}\left(t\right)w_{jt}^{\alpha }K\left(x_{i},z_{j}\right)+\beta f_{y}\left(t\right)w_{jt}^{\alpha }K\left(y_{i},z_{j}\right)\right]}. \end{array}$$

Therefore, an optimized FCM algorithm based on anisotropic filtering can be obtained, which is set as AFFCM. The calculation process is shown in Figure 1. First, the FCM algorithm's parameters are initialized, the image is preprocessed by anisotropic filtering, and the histogram function of the original image and the filtered image is obtained. Then, the membership matrix and clustering center are calculated and updated. If *t* ≤ *T*, the algorithm ends. Otherwise, the above steps are repeated. Finally, the image is deblurred to judge the categories of image elements.

### 2.4. Evaluation Criteria for Image Segmentation

The traditional FCM algorithm, KFCM [13], and RFCM [14] were introduced for comparison with AFFCM constructed in this study. Moreover, the results of image segmentation were evaluated by using three indicators of correlation degree between classes after fuzzy, partition coefficient, and segmentation entropy, which could be calculated as follows:

(19) $$\begin{array}{c} Q_{pc}=\frac{\sum_{i=1}^{s}\sum_{j=1}^{n}w_{ij}^{2}}{n}. \end{array}$$

(20) $$\begin{array}{c} Q_{pe}=-\frac{\sum_{i=1}^{s}\sum_{j=1}^{n}\left(w_{ij}\log\;w_{ij}\right)}{n}. \end{array}$$

(21) $$\begin{array}{c} Q_{da}=-\frac{\sum_{j=1}^{s}\sum_{j=1}^{n}w_{ij}{\left\|x_{j}-z_{i}\right\|}^{2}}{n\left(\min i\neq k\left\|z_{k}-z_{i}\right\|\right)}. \end{array}$$

In equations (19), (20), and (21), *Q*_*pc*_ represented the partition coefficient, *Q*_*pe*_ stood for the segmentation entropy, *Q*_*da*_ meant the correlation degree between classes after fuzzy, and the other letters had the same meaning as above. When performing image segmentation, the larger the value *Q*_*pc*_, the better the segmentation effect; the smaller the value *Q*_*pe*_, the better the segmentation effect; the smaller the value *Q*_*da*_, the better the segmentation effect.

### 2.5. Observation Indicators

Three indicators of AFFCM, FCM, KFCM, and RFCM needed to be recorded, which were the partition coefficient, segmentation entropy, and the correlation degree between classes after fuzzy. Then, the location and distribution of foreign bodies in the trachea and the types of foreign bodies should be collected. MRI scanning and chest X-ray were recorded for the diagnosis of tracheal foreign body (positive and negative), and the positive rate of diagnosis was calculated. In addition, the indirect signs of tracheal foreign bodies in the children were recorded by MRI scanning and chest X-ray.

### 2.6. Statistical Methods

SPSS 19.0 statistical software was used for test data processing, the measurement data were expressed as the mean ± standard deviation ($\bar{x}$ ± s), the count data were represented by percentage (%), and the AFFCM, FCM, KFCM, and RFCM were compared by one-way analysis of variance (ANOVA). Furthermore, MRI scanning and X-ray chest radiographs adopted *t*-test to compare the positive rate and the diagnosis rate of tracheal foreign bodies in children, and *P* < 0.05 indicated that the difference was statistically marked.

## 3. Results

### 3.1. Comparison on the Segmentation Performance of Different Algorithms

Figure 2 reveals that the partition coefficient and the correlation degree between classes after fuzziness of AFFCM increased greatly in contrast to those of FCM, KFCM, and RFCM, with a statistically marked difference (*P* < 0.05). The segmentation entropy of AFFCM (0.137) was smaller steeply than the entropies of FCM (0.447), KFCM (0.322), and RFCM (0.275), and there was a statistically obvious difference (*P* < 0.05). The partition coefficient and the correlation degree between classes after fuzziness of KFCM (0.347) and RFCM (0.406) were markedly greater than those of FCM (0.288) (*P* < 0.05), while the segmentation entropies of KFCM and RFCM were both hugely smaller than that of FCM (*P* < 0.05).

Figure 3 shows the comparison of MRI images processed by different algorithms. It was found that the original image map had poor clarity and more artifacts and noises, and the observation of image features was not clear enough, with poor quality. After the four algorithms, the sharpness of the image was improved to a certain extent, and the noise was correspondingly reduced. Among them, the sharpness of the image processed by AFFCM was the highest, with less noise and artifacts, and the quality was improved hugely.

### 3.2. X-Ray and MRI Imaging Evaluation of One Child Patient

Figure 4 shows the X-ray and MRI image evaluation of one case (male, 2 years old). X-ray film revealed that the transmittance of the left lung field decreased, the mediastinum moved to the left, the transmittance of the right lung field increased, the air content rose, and there were obvious manifestations of emphysema. Considering the valve function of the foreign body, the volume of air inhaled was more than the volume of air exhaled, resulting in the increased volume of air in the right lung and emphysema, so he was diagnosed as a right bronchial foreign body. The right lung emphysema could be observed from the MRI image, the T1-weighted image was an iso-signal shadow, and the T2-weighted image was a high-intensity shadow. Thus, the diagnosis was a vegetative bronchial foreign body.

### 3.3. The Situation of Foreign Bodies in the Bronchus of 28 Child Patients

Figure 5 reveals that there were 5 cases of foreign bodies in the trachea (17.86%), 10 cases of foreign bodies in the left bronchus (35.71%), and 13 cases of foreign bodies in the right bronchus (46.43%) among the 28 child patients.

As for the types of foreign bodies, 10 cases were melon seeds (35.71%), 6 cases were peanuts (21.43%), 5 cases were beans (17.86%), 3 cases were pistachios (10.71%), 3 cases were plastic (10.71%), 1 case was fish bone (3.57%), most of which were plant-based foreign bodies, as shown in Figure 6.

### 3.4. Comparison on Positive Rate and Diagnosis Rate of MRI and X-Ray Diagnosis of Bronchial Foreign Bodies

Figure 7 discloses the comparison results of the positive rates of MRI and X-ray diagnosis of bronchial foreign bodies. It was found that MRI diagnosis of bronchial foreign bodies was positive in 25 cases and negative in 3 cases; chest X-ray diagnosis of bronchial foreign bodies was positive in 16 cases and negative in 12 cases. The positive rate of MRI diagnosis of bronchial foreign bodies (89.29%) rose substantially compared with X-ray chest radiograph (57.14%), and the difference was obvious (*P* < 0.05). Besides, the negative rate of MRI diagnosis of bronchial foreign bodies (10.71%) dropped sharply in contrast to the rate of X-ray chest radiograph (42.86%), showing a statistically huge difference (*P* < 0.05).

The diagnosis rates of MRI and X-ray diagnosis of tracheal foreign bodies were compared, and the results are presented in Figure 8. It shows that the diagnosis rate of tracheal foreign bodies diagnosed by MRI (96.43%) elevated obviously compared with chest X-ray (67.96%) (*P* < 0.05). However, the negative diagnosis rate of tracheal foreign bodies diagnosed by MRI (3.57%) reduced steeply in contrast to the rate of chest X-ray (32.14%) (*P* < 0.05).

### 3.5. MRI and X-Ray Diagnosis of Tracheal Foreign Body Signs

Figure 9 displays the signs of foreign bodies in trachea diagnosed by MRI and X-ray. It reveals that the X-ray diagnosis of bronchial foreign body signs included emphysema, atelectasis, limited obstruction, and mediastinal displacement. Among them, 21 child patients suffered from emphysema, 8 child patients had atelectasis, 1 child patient suffered from limited obstruction, and 2 child patients showed mediastinal displacement; thus emphysema > atelectasis > mediastinal displacement > limited obstruction. The bronchial foreign body signs diagnosed through MRI were emphysema, atelectasis, mediastinal swing, limited obstruction, mediastinal displacement, and pulmonary infection. Among them, there were 25 cases with emphysema, 22 cases with atelectasis, 17 cases with mediastinal swing, 10 cases with limited obstruction, 3 cases with mediastinal displacement, and 19 cases with pulmonary infection, so emphysema > atelectasis > pulmonary infection > mediastinal swing > limited obstruction > mediastinal displacement.

## 4. Discussion

Tracheal and bronchial foreign bodies refer to the symptoms of coughing, wheezing, and dyspnea caused by foreign bodies entering the respiratory tract through inhalation, ingestion, suffocation, and so forth. Kozaci et al. (2019) [15] found that when a foreign body entered the human airway, it would stimulate the airway mucosa and cause mucosal edema. If it stayed in the airway for too long, it would also lead to pneumonia and lung abscess. Therefore, it is necessary to choose an accurate way to diagnose and treat airway foreign bodies. MRI, as an imaging method extensively used in the field of medical diagnosis in recent years, has very prominent advantages, but it is rarely applied in the diagnosis of foreign bodies in the trachea. In this study, the traditional FCM algorithm was first optimized based on anisotropic filtering (AFFCM), which was compared with FCM, KFCM, and RFCM. The result indicated that the partition coefficient and the correlation degree between classes after fuzziness of AFFCM were hugely greater than those of FCM, KFCM, and RFCM, but the segmentation entropy of AFFCM was obviously smaller than those of FCM, KFCM, and RFCM (*P* < 0.05). This was similar to the research findings of Tamiru et al. (2012) [16], which showed that, compared with the traditional algorithm, the proposed algorithm AFFCM had higher segmentation coefficient value, lower segmentation entropy, higher similarity between classes, and better image segmentation effect [17]. Based on the processed MRI images, AFFCM could overcome noise and improve image quality.

In this study, MRI and X-ray scanning based on AFFCM were performed on 28 children who were diagnosed with tracheal foreign bodies and admitted to the hospital from October 2019 to November 2020. It was found that there were 5 cases (17.86%) of tracheal foreign bodies, 10 cases (35.71%) of left bronchial foreign bodies, and 13 cases (46.43%) of right bronchial foreign bodies in the 28 children, which was consistent with previous studies, showing that the right bronchial foreign body was the most common site. Among the 28 cases of foreign bodies, 10 cases were melon seeds (35.71%), 6 cases were peanuts (21.43%), 5 cases were beans (17.86%), and other types were few, most of which were plant foreign bodies. This may be due to the fact that melon seeds are always available in every family. When children are frightened, crying, and naughty, and there are other predisposing factors, it is easy to accidentally choke into the airway [18]. The positive rate (89.29%) and diagnosis rate (96.43%) of bronchial foreign body diagnosed by MRI were substantially higher than the rates of chest X-ray (57.14% and 67.86%) (*P* < 0.05), which was similar to the research findings of Gao et al. (2015) [19], indicating that the diagnostic level of coronal MRI for airway foreign bodies was better than that of chest X-ray film. What is more, it could clearly show the size, shape, and type of foreign bodies as well as the complications caused to the lungs, and it was easier to identify the related diseases. The bronchial foreign body signs through MRI diagnosis were emphysema > atelectasis > lung infection > mediastinal swing > limited obstruction > mediastinal displacement, in which emphysema and atelectasis were the most common cases, suggesting that emphysema and atelectasis could be the main signs of bronchial foreign body in MRI diagnosis. In the X-ray diagnosis of bronchial foreign body signs, emphysema > atelectasis > mediastinal displacement > limited obstruction, where the number of emphysema cases was the largest, which indicated that emphysema could be used as the primary sign of X-ray diagnosis of bronchial foreign bodies.

## 5. Conclusion

In this study, the traditional FCM algorithm was optimized based on anisotropic filtering to obtain AFFCM, and it was compared with FCM, KFCM, and RFCM, which was also applied to 28 cases of pediatric tracheal foreign body MRI diagnosis. It was found that AFFCM had a relatively high partition coefficient value, a lower segmentation entropy, and a greater degree of similarity between classes, with better image segmentation effect. MRI based on AFFCM also had a higher positive rate and diagnosis rate for children with foreign bodies in the trachea, and the main signs were emphysema and atelectasis. However, the selection of children's samples is small in this study, and more detailed group discussions are not possible. Further consideration is given to the selection of more children to further explore the characteristics of tracheal foreign body in MRI images of child patients. All in all, the results of this study can provide a good theoretical basis for the clinical diagnosis of foreign bodies in the trachea of children.

## Figures and Tables

**Figure 1:** Algorithm's flow chart.

**Figure 2:** Comparison on partition coefficients, segmentation entropy, and the correlation degree between classes after fuzziness of different algorithms: (a) the partition coefficient; (b) the segmentation entropy; (c) the correlation degree between classes after fuzziness. *∗* indicates *P* < 0.05 compared with AFFCM; # indicates *P* < 0.05 compared with FCM.

**Figure 3:** Comparison on the segmentation performance of different algorithms: (a) the original image; (b) the image processed by FCM; (c) the image processed by KFCM; (d) the image processed by RFCM; and (e) the image processed by AFFCM constructed in this study.

**Figure 4:** X-ray and MRI image evaluation of a male case (2 years old): (a) a chest X-ray; (b) an MRI image.

**Figure 5:** The distribution of foreign bodies in the bronchus of 28 child patients: 1: the foreign bodies in the trachea; 2: the foreign bodies in the left bronchus; 3: the foreign bodies in the right bronchus.

**Figure 6:** Types of bronchial foreign bodies in 28 child patients.

**Figure 7:** Comparison on positive rates of MRI and X-ray diagnosis of bronchial foreign bodies: *∗* indicates *P* < 0.05 by comparison with MRI.

**Figure 8:** Comparison of the diagnosis rates of MRI and X-ray diagnosis of tracheal foreign bodies: *∗* indicates *P* < 0.05 compared to MRI.

**Figure 9:** Comparison of the tracheal foreign body signs of MRI and X-ray diagnosis: *∗* indicates *P* < 0.05 compared with X-ray.

## Data Availability

No data were used to support this study.
